The article "The potency of lncRNA MALAT1/miR-155/CTLA4 axis in altering Th1/Th2 balance of asthma" was retracted in 2023. Reasons: duplicated images; concerns about the images.

# The potency of lncRNA MALAT1/miR-155/CTLA4 axis in altering Th1/Th2 balance of asthma

**DOI:** 10.1042/BSR20190397

**Published:** 2020-02-14

**Authors:** Zhijun Liang, Fenglian Tang

**Affiliations:** Department of Respiratory Medicine, Affiliated Hospital of Jining Medical University, Jining City 272000, Shandong Province, China

**Keywords:** asthma, CTLA-4, lncRNA MALAT1, miR-155, T-bet/Gata3 ratio, Th1/Th2 balance

## Abstract

**Objectives:** The present study examined if the metastasis-associated lung adenocarcinoma transcript 1 (MALAT1)/miR-155/CTLA-4 axis was involved in modifying Th1/Th2 balance, a critical indicator for asthma progression. **Methods:** Altogether 772 asthma patients and 441 healthy controls were recruited, and their blood samples were collected to determine expressional levels of MALAT1, miR-155, CTLA-4, T-bet, GATA3, Th1-type cytokines and Th2-type cytokines. The CD^4+^ T cells were administered with pcDNA3.1-MALAT1, si-MALAT1, miR-155 mimic and miR-155 inhibitor to assess their effects on cytokine release. The luciferase reporter gene assay was also adopted to evaluate the sponging relationships between MALAT1 and miR-155, as well as between miR-155 and CTLA-4. **Results:** Over-expressed MALAT1 and under-expressed miR-155 were more frequently detected among asthma patients who showed traits of reduced forced expiratory failure volume in 1 s (FEV1), FEV1/forced vital capacity (FVC) and FEV1% of predicted (*P*<0.05). Moreover, MALAT1 expression was negatively expressed with the Th1/Th2 and T-bet/GATA3 ratios, yet miR-155 expression displayed a positively correlation with the ratios (*P*<0.05). Additionally, the IFN-γ, IL-2 and T-bet levels were reduced under the influence of pcDNA3.1-MALAT1 and miR-155 inhibitor, while levels of IL-4, IL-10 and GATA3 were raised under identical settings (*P*<0.05). Furthermore, MALAT1 constrained expression of miR-155 within CD^4+^ T cells by sponging it, and CTLA-4 could interfere with the effects of MALAT1 and miR-155 on Th1/Th2 balance and T-bet/Gata3 ratio (*P*<0.05). **Conclusion:** MALAT1 sponging miR-155 was involved with regulation of Th1/Th2 balance within CD^4+^ T cells, which might aid to develop therapies for amelioration of asthmatic inflammation.

## Introduction

Bronchial asthma, a chronic inflammatory disorder, is clinically manifested as recurrent wheezing, chest distress and cough [1,2]. According to the estimation of World Health Organization (WHO), the global prevalence of asthma has reached up to 300 million, and delayed treatments could increase disease mortality [3,4]. Multiple factors induce asthma, including environment, heredity and immunity [5,6]. Of note, one immunity-centric theory proposed that asthmatic progression was accompanied by Th2-oriented differentiation of T lymphocytes, and the latter favored release of Th2-type cytokines over production of Th1-type cytokines [7,8]. The resultant bias of Th1/Th2 ratio was a trigger of dysfunctional cell immunity and humoral response, which finally led to asthma exacerbation [9,10]. From the above, suppressing T-cell activation or elevating the Th1/Th2 ratio might be conducive to relieving asthma-relevant inflammation from the source.

The article "The potency of lncRNA MALAT1/miR-155/CTLA4 axis in altering Th1/Th2 balance of asthma" was retracted in 2023. Reasons: duplicated images; concerns about the images.

LncRNAs, molecules with a length of more than 200 nucleotides, regulate numerous biological processes in humans [11,12]. The crucial role of lncRNAs in modulating asthma development has also been increasingly stressed, given their involvement in regulating the inflammatory mechanism [13,14] and function of airway smooth muscle (ASM) [15–17]. For instance, lipopolysaccharide (LPS)-induced inflammation is enhanced after knockout of lncRNA interleukin 7 receptor (IL7R) [13], and expression of lncRNA H19 was reduced after stimulation of pro-inflammatory cytokines (e.g. IL-1β and TNF-α) [18]. On the other hand, exposure to fetal calf serum (FCS) and dexamethasone was found to engender expressional changes of LINC00882, LINC00883 and lncRNA PVT1 within ASM cells (ASMCs) [15]. Notably, the lncRNA metastasis-associated lung adenocarcinoma transcript 1 (MALAT1) investigated here was also potentially relevant to asthma etiology, owing to MALAT1 that was able to aggravate inflammatory reactions via negative modification of miR-125b [19]. MiR-125b was markedly under-expressed within asthma patients when compared with healthy controls, and it was a sensitive reflector of asthma severity [20]. In addition, under-expression of MALAT1 was discovered to ease symptoms of myocardial inflammation [21], and production of TNF-α and IL-6 in endothelial cells was spurred when MALAT1 expression was intentionally elevated [22,23]. These findings all indicated that MALAT1 was associated with activation of inflammation, though whether MALAT1 indeed affected asthma-related inflammation remained unknown.

Additionally, miRNAs are commonly acknowledged collaborators of lncRNAs in precise regulation of disease pathogenesis [24], and they are also indispensable modulators for certain inflammatory airway diseases (e.g. asthma) [25]. For instance, the expressional range of miR-155, which was sponged by MALAT1 [26], could mirror evolution of airway inflammation and airway hyper-responsiveness that occurred in ovalbumin (OVA)-sensitized asthmatic mice [27–29]. The intrinsic mechanism might be due to the fact that miR-155 regulated differentiation of T cells (e.g. Th2, Th17 and Treg cells) [30–33] and the antigen-presenting process of dendritic cells (DCs) [34–36]. More than that, certain genes (e.g. *CTLA-4*) were capable assistants of miR-155 in changing the activity of Th cells and thereby in inducing asthma onset [37]. Nevertheless, further data were needed to determine whether MALAT1 combined with miR-155 and CTLA-4 could drive the onset of asthma.

The article "The potency of lncRNA MALAT1/miR-155/CTLA4 axis in altering Th1/Th2 balance of asthma" was retracted in 2023. Reasons: duplicated images; concerns about the images.

To tentatively tap this field, we attempted to figure out if MALAT1 was capable of altering Th1/Th2 balance in the context of asthma, which might offer a novel direction for preventing asthmatic inflammation.

## Materials and methods

### Inclusion of study subjects

From April 2015 to May 2018, we recruited 772 asthma patients from Affiliated Hospital of Jining Medical University, and they all met the diagnostic criteria for acute attack of asthma [38]. The asthma patients all showed no liver or kidney-related dysfunctions, and they were not plagued by respiratory tract infection (RTI) or heart failure within the past 2 months. Simultaneously, 441 healthy volunteers were incorporated into the control group, and none of them carried infectious disorders within the past 2 months. All the participants signed informed consents, and procedures of this investigation gained approval from Affiliated Hospital of Jining Medical University and the Ethics Committee of Affiliated Hospital of Jining Medical University.

### Evaluation of Th1/Th2 balance among asthma patients

Approximately 5 ml venous blood was collected from each asthma patient, and the blood samples were centrifuged at 16000×***g*** for 10 min to acquire the supernatants. Then expressions of Th1-type cytokines (i.e. IL-2 and IFN-γ) and Th2-type cytokines (i.e. IL-4 and IL-10) were measured according to the guidance of respective enzyme-linked immuno-sorbent assay (ELISA) kits (ZSBIO, Beijing, China), and the Th1/Th2 ratio was calculated as per the formula of (Concentration_IL-2_ + Concentration_IFN-_γ)/(Concentration_IL-4_ + Concentration_IL-10_). Moreover, expressions of T-bet and GATA3 were evaluated through performing Western blotting as specified below, and expressions of MALAT1 and miR-155 were determined by means of reverse transcription-polymerase chain reaction (RT-PCR) also as depicted below. All these experiments were repeated for more than or equal to three times.

### Separation of CD^4+^ T cells

Approximately 5 ml peripheral blood was gathered from healthy volunteers, with ethylene diamine tetraacetic acid (EDTA)-K2 added in advance for anti-coagulation. Then, peripheral blood mononuclear cells (PBMCs) were isolated under the weight of lymphocyte separation medium (Sangon, China). After rinsing the PBMCs with phosphate buffer (PBS) for twice, the CD^4+^ T cells were separated through a magnetic activated cell sorting (MACS) system (Miltenyi Biotech, German). The specific procedures were summarized as: (1) every 1 × 10^8^ cells were mixed with 900 μl solution that was composed of 2 mmol/l EDTA, 20 ml/l FBS and PBS; (2) 100 μl of CD^4^ microbeads (Miltenyi Biotech, German) were supplemented proportionally; (3) incubation was sustained in the dark for 20 min, followed by rinse of LS column with 3 ml of solution; (4) 1000 rpm centrifugation was performed for 10 min after addition of 10 ml of solution; (5) the resultant supernatants were removed before re-suspension of cell sediments in 2 ml of solution; (6) the cells that dropped from MACS were CD^4−^ T cells; (7) LS column was transferred on to the centrifugal tube and was washed with 5 ml of solution; and (8) the cells finally collected were CD^4+^ T cells. All these experiments were repeated for more than or equal to three times.

The article "The potency of lncRNA MALAT1/miR-155/CTLA4 axis in altering Th1/Th2 balance of asthma" was retracted in 2023. Reasons: duplicated images; concerns about the images.

### Western blotting

The serum and cells were centrifuged at 12000×***g*** for 15 min, after being mixed with radio-immunoprecipitation assay (RIPA) lysis buffer and pre-cooled 10% phenylmethanesulfonyl fluoride (PMSF). Then the collected supernatants were blended with 5× sampling buffer, before being boiled for 5 min. Subsequently, the resultants were prepared to undergo 10% sodium dodecyl sulphate/polyacrylamide gel electrophoresis (SDS/PAGE), after which the mixture was transferred on to the polyvinylidene fluoride (PVDF) membrane. After 1-h blockage with 5% skimmed milk at room temperature, the primary antibodies (Abcam, U.S.A.) against IFN-γ (mouse anti-human, 1:500, Cat. No.: ab9801), IL-2 (rabbit anti-human, 1:1000, Cat. No.: ab180780), T-bet (mouse anti-human, 1:1000, Cat. No.: ab91109), IL-4 (mouse anti-human, 1:500, Cat. No.: 34277), IL-10 (rabbit anti-human, 1:2000, Cat. No.: ab34843), GATA3 (rabbit anti-human, 1:1000, Cat. No.: 199428), CTLA-4 (rabbit anti-human, 1:5000, Cat. No.: 134090), GAPDH (rabbit anti-human, 1:2500, Cat. No.: 9485) and β-actin (rabbit anti-human, 1:1000, Cat. No.: 8226) were supplemented for overnight incubation. With Tris-Buffered Saline Tween (TBST) adopted to rinse the products for three times, corresponding goat anti-mouse secondary antibodies labeled by horseradish peroxidase (HRP) were additionally prepared to incubate the mixture for 1 h. Eventually, development was fulfilled utilizing electro-chemi-luminescence (ECL) (Amershan Biosciences, Sweden), and AlphaEaseFCTM software was employed to analyze the protein bands. All these experiments were repeated for more than or equal to three times.

### RT-PCR

Total RNA was extracted from serum and CD^4+^ T cells with aid of TRizol reagent (TIANGEN, China), and its integrity was confirmed by PAGE. The quality of total RNA was deemed as desirable if the A260/A280 ratio drawn from ultraviolet spectrophotometry ranged between 1.8 and 2.1. Afterward, the total RNAs were reversely transcribed into cDNAs by feat of PrimeScript™ RT reagent kit (TaKaRa, Japan), and PCR was accomplished on a real-time PCR instrument (model: LightCycler 480®, Roche, Switzerland), according to specifications indicated in the SYBR Premix Ex Taq™ kit (TaKaRa, Japan). Aided by primers (Table 1) that were designed via Primer 5.0 software and synthesized by Sangon (China), the aforementioned PCR was implemented under conditions of: (1) pre-denaturation at 95°C for 30 s as well as (2) 40 cycles of denaturation at 95°C for 5 s, renaturation at 63°C for 30 s and extension at 95°C for 10 s. Finally, expressions of target genes were quantified in line with the 2^−ΔΔ*C*_t_^ method, with GAPDH and U6, respectively, set as the internal reference for MALAT1 and miR-155. All these experiments were repeated for more than or equal to three times.

The article "The potency of lncRNA MALAT1/miR-155/CTLA4 axis in altering Th1/Th2 balance of asthma" was retracted in 2023. Reasons: duplicated images; concerns about the images.

**Table 1:** Primer sequences used in real-time PCR are written in 5′–3′ direction

Gene	Primers	
	Forward	Reverse
*MALAT1*	AAGATGAGGGTGTTTACG	AAGCCTTCTGCCTTAGTT
*miR-155*	CTCGTGGTTAATGCTAATTGTGA	GTGCAGGGTCCGAGGT
*CTLA-4*	AACCTTCAGTGGTGTTGGCTA	GTCATTTGGTCATTTGTCTGC
*IFN-γ*	AGTTATATCTTGGCTTTTCA	ACCGAATAATTAGTCAGCTT
*IL-2*	AACTCCTGTCTTGCATTGCACTA	TTGCTGATTAAGTCCCTGGGTC
*T-bet*	GTGACCCAGATGATTGTGCTC	GTAGGCAGTCACGGCAATG
*IL-4*	CTTCCCCCTCTGTTCTTCCT	TTCCTGTCGAGCCGTTTCAG
*IL-10*	ATGCCCCAAGCTGAGAACCAAGACCCA	TCTCAAGGGGCTGGGTCAGCTATCCCA
*GATA3*	ATGGCACGGGACACTACCT	TCCCCATTGGCATTCCTC
*GAPDH*	GGTTGTCTCCTGCGACTTCA	TGGTCCAGGGTTTCTTACTCC
*U6*	CTCGCTTCGGCAGCACA	AACGCTTCACGAATTTGCGT
*β-actin*	CCAGTGGACATCGCCAAAGACG	TCCAAGAAAGCGGTGTAACCAGAC

### Cell transfection and treatment

The pcDNA3.1-MALAT1 and siRNAs interfering with MALAT1 (i.e. siMALAT1-1: 5′-GCCGAAATAAATGAGAGATGA-3′; siMALAT1-2: 5′-GGCAGCTGTTAACAGATAAGT-3′; siMALAT1-3: 5′-GCTGTGGAGTTCTTAAATATC-3′; siMALAT1-4: 5′-GGGCTTCAGTGATGGGATAGT-3′) were designed and synthesized by Genechem (China). In addition, miR-155 inhibitor (5′-ACCCCUAUCACGAUUAGCAUUAA-3′), miR-155 mimic (sense: 5′-UUAAUGCUAAUUGUGAUAGGGGU-3′, antisense: 5′-CCCUAUCACAAUUAGCAUUAAUU-3′). and miR-NC (5′-UCUACUCUUUCUAGGAGGUUGUGG-3′) were provided by GenePharma (China), and siRNAs of CTLA-4 (si-CTLA4-1, sense: 5′-CCCAAAUUACGUGUACUAC-3′, antisense: 5′-GUAGUACACGUAAUUUGGG-3′; si-CTLA4-2, sense: 5′-CGGAACCCAGAUUUAUGUA-3′, antisense: 5′-UACAUAAAUCUGGGUUCCG-3′; si-CTLA4-3, sense: 5′-GGUGGAGCUCAUGUACCCA-3′, antisense: 5′-UGGGUACAUCAGCUCCACC-3′) and pcDNA3.1-CTLA4 were also prepared in advance. The pcDNA3.1-MALAT1, si-MALAT1, miR-155 mimic, miR-155 inhibitor, miR-NC, si-CTLA4 and pcDNA3.1-CTLA4 were then, respectively, transfected into CD^4+^ T cells, following the guidance of Lipfectamine™ 2000 kit (Invitrogen, U.S.A.). The abovementioned experiments were duplicated for more than or equal to three times.

The article "The potency of lncRNA MALAT1/miR-155/CTLA4 axis in altering Th1/Th2 balance of asthma" was retracted in 2023. Reasons: duplicated images; concerns about the images.

### Dual-luciferase reporter gene assay

The MALAT1 and CTLA-4 fragments that contained target sites of miR-155 were amplified through conduction of PCR. The products were then cloned into pRL-TK/Rluc plasmids (Promega, U.S.A.) to establish pRL-TK/Rluc-MALAT1 wild-type (Wt) and pRL-TK/Rluc-CTLA-4 Wt. The pRL-TK/Rluc-MALAT1 mutant type (Mut) and pRL-TK/Rluc-CTLA-4 Mut were produced analogously, except that MALAT1 and CTLA-4 fragments were mutated in their miR-155-binding sites. Subsequently, pRL-TK/Rluc-MALAT1 Wt, pRL-TK/Rluc-CTLA-4 Wt, pRL-TK/Rluc-MALAT1 Mut and pRL-TK/Rluc-CTLA-4 Mut were, respectively, co-transfected with miR-155 mimic or miR-NC into CD^4+^ T cells, according to the instructions of Lipofectamine ™ 2000 kit (Invitrogen, U.S.A.). Approximately 48 h later, the luciferase activity was detected on the dual-luciferase® reporter assay system (Promega, U.S.A.). All these experiments were repeated for more than or equal to three times.

### Statistical analyses

All the statistical analyses were implemented with usage of SPSS software v17.0 and GraphPad Prism v5. The measurement data, which were manifested as mean ± standard deviation (SD), were compared based on Student’s *t* test or analysis of variance (ANOVA). The categorical data in the form of *n* or percentage (%) were analyzed by adopting chi-square test. It was regarded as statistically significant in case that *P*-value was less than 0.05.

## Results

### Association of MALAT1/miR-155 expression with clinical traits of asthma patients

The asthma patients and healthy controls were well matched in their mean age, sex ratio, body mass index (BMI) and smoking history (*P*>0.05) and, as expected, a higher proportion of asthma history was observed among asthma patients when compared with healthy controls (χ^2^ = 10.72, *P*=0.001) (Table 2). Moreover, production of fractional exhaled nitric oxide (FeNO) was greater in asthma subjects as compared with healthy people (*P*<0.05). The healthy population had a higher forced expiratory failure volume in 1 s (FEV1), FEV1/forced vital capacity (FVC) and FEV1% of predicted when compared with asthma patients (*P*<0.05). In addition, differential expressions of MALAT and miR-155 were also observed between asthma patients and healthy controls (*P*<0.05) (Figure 1A). With median MALAT1 expression as the dividing line, the recruited asthma patients were grouped into those with highly expressed MALAT1 and those carrying lowly expressed MALAT1. In the same manner, the highly expressed (>median) miR-155 group and lowly expressed (≤median) miR-155 group were also drawn from the identical asthma group (Table 3). It was interesting to observe that the asthma patients who carried lowly expressed MALAT1 and highly expressed miR-155 were more prone to reveal higher FEV1 (>1.95 l), FEV1/FVC (>71.55%), predicted FEV1% (>78.91%) and FeNO (≤51.27 μg/l) than highly expressed MALAT1 group and lowly expressed miR-155 group (*P*<0.05).

The article "The potency of lncRNA MALAT1/miR-155/CTLA4 axis in altering Th1/Th2 balance of asthma" was retracted in 2023. Reasons: duplicated images; concerns about the images.

**Table 2:** Comparison of clinical features between asthmatic patients and healthy controls

Clinical features	Asthmatic patients	Healthy controls	t/χ^2^	*P*-value
Age (years)	49.68 ± 13.31	50.85 ± 15.64	1.38	0.168
Gender				
Female	449	234		
Male	323	207	2.97	0.085
BMI (kg/m^2^)	26.71 ± 5.52	26.05 ± 6.46	1.88	0.060
Smoking				
Yes	315	156		
No	457	285	3.483	0.062
Asthma history				
Yes	342	153		
No	430	288	10.72	0.001
FEV1 (l)	1.95 ± 0.78	2.54 ± 0.63	13.56	<0.001
FEV1/FVC (%)	71.55 ± 5.46	89.61 ± 3.12	63.76	<0.001
FEV1% of predicted	78.91 ± 5.33	97.53 ± 3.68	65.03	<0.001
FeNO (μg/l)	51.27 ± 5.39	23.86 ± 4.51	90.25	<0.001

**Figure 1:** Correlation of lncRNA MALAT1 and miR-155 with Th1/Th2 balance and T-bet/GATA3 ratio among asthma patients (**A**) Expressions of MALAT1 and miR-155 were compared between asthma patients and healthy controls. *: *P*<0.05 when compared with healthy control. (**B**) Expressions of T-bet and GATA3 were detected among asthma patients and healthy controls. *: *P*<0.05 when compared with healthy control. (**C**) Expression of MALAT1 was negatively associated with Th1/Th2 and T-bet/GATA3 among the incorporated asthma patients. (**D**) The expression of miR-155 was positively correlated with Th1/Th2 and T-bet/GATA3 ratios among asthma patients. (**E**) There showed a positive correlation between Th1/Th2 ratio and T-bet/GATA3 ratio among asthma patients.

**Table 3:** Association of lncRNA MALAT1 and miR-155 expressions with baseline characteristics of asthmatic patients

Clinical features	LncRNA MALAT1 expression				miR-155 expression			
	Low	High	χ^2^	*P*-value	Low	High	χ^2^	*P*-value
Age (years)								
>49.68	151	243			212	182		
≤49.68	136	242	0.45	0.500	211	167	0.32	0.574
Gender								
Female	173	276			255	194		
Male	114	209	0.84	0.359	168	155	1.73	0.188
BMI (kg/m^2^)								
>26.71	134	241			214	161		
≤26.71	153	244	0.65	0.42	209	188	1.52	0.217
Smoking								
Yes	118	197			178	137		
No	169	288	0.02	0.892	245	212	0.63	0.427
Asthma history								
Yes	116	226			194	148		
No	171	259	2.79	0.095	229	201	0.93	0.336
FEV1 (l)								
>1.95	153	217			188	182		
≤1.95	134	268	5.30	0.021	235	167	4.55	0.033
FEV1/FVC (%)								
>71.55	180	241			204	217		
≤71.55	107	244	12.34	<0.001	219	132	15.01	<0.001
FEV1% of predicted								
>78.91	168	235			199	204		
≤78.91	119	250	7.35	0.007	224	145	9.97	0.002
FeNO (μg/l)								
>51.27	130	266			237	159		
≤51.27	157	219	6.58	0.010	186	190	8.39	0.004

The article "The potency of lncRNA MALAT1/miR-155/CTLA4 axis in altering Th1/Th2 balance of asthma" was retracted in 2023. Reasons: duplicated images; concerns about the images.

### Links of MALAT1/miR-155 expression with Th1/Th2 balance and T-bet/GATA3 ratio among the included asthma patients

Expression of Th1-type cytokines (i.e. IL-2 and IFN-γ) and T-bet were significantly reduced in asthma patients when compared with healthy controls, which ran counter to the expressional tendency of Th2-type cytokines (i.e. IL-4 and IL-10) and GATA3 (*P*<0.05) (Table 4). Also, either Th1/Th2 ratio or T-bet/GATA3 ratio observably dropped in the asthma group, as compared with the control group (*P*<0.05) (Figure 1B). In addition, MALAT1 expression was down-regulated and miR-155 expression was up-regulated, along with the ascent of Th1/Th2 ratio (MALAT: r_s_ = −0.346, miR-155: r_s_ = 0.362) and T-bet/GATA3 ratio (MALAT: r_s_ = −0.368, miR-155: r_s_ = 0.335) (Figure 1C,D). There also was a positive correlation between the T-bet/GATA3 ratio and Th1/Th2 ratio among the recruited asthma patients (r_s_ = 0.395, *P*<0.001) (Figure 1E).

**Table 4:** Comparison of cytokine levels among asthmatic patients at the acute stage, asthmatic patients at the remission stage and healthy controls

Cytokines	Healthy control	Asthmatic patients
*Th1-related cytokine*		
IL-2 (ng/l)	254.8 ± 54.16	181.20 ± 57.94*
IFN-γ (ng/l)	67.29 ± 8.87	46.21 ± 17.36*
*Th2-related cytokine*		
IL-4 (ng/l)	56.81 ± 16.48	111.56 ± 48.73*
IL-10 (ng/l)	29.31 ± 7.62	60.55 ± 26.80*
Th1/Th2	3.47 ± 0.81	1.48 ± 0.66*
T-bet	1.00 ± 0.04	0.37 ± 0.09*
GATA3	1.00 ± 0.05	1.90 ± 0.22*
T-bet/GATA3	1.91 ± 0.65	0.26 ± 0.09*

* The *P*-value ≤ 0.05 when compared with healthy control.

### MALAT1 and miR-155 affected Th1/Th2 balance and T-bet/Gata3 ratio in CD^4+^ T cells

Expression of MALAT1 was evidently promoted within CD^4+^ T cells of pcDNA3.1-MALAT1 group (*P*<0.05), yet it was down-regulated greatly under the weight of si-MALAT1-1, si-MALAT1-2, si-MALAT1-3 and si-MALAT1-4 (*P*<0.05) (Figure 2A). In addition, exposure to miR-155 mimic and miR-155 inhibitor, respectively, raised and lessened expression of miR-155 within CD^4+^ T cells (*P*<0.05) (Figure 2B). Moreover, both under-expressed MALAT1 and over-expressed miR-155 could spur production of IFN-γ, IL-2 and T-bet (*P*<0.05), which were, on the contrary, repressed under the action of over-expressed MALAT1 and under-expressed miR-155 (*P*<0.05) (Figure 2C,D). Correspondingly, the mRNA and protein levels of IL-4, IL-10 and GATA3 were heightened within CD^4+^ T cells of the pcDNA3.1-MALAT1 group and the miR-155 inhibitor group, though they were lowered within CD^4+^ T cells of the si-MALAT1-3 group and the miR-155 mimic group (*P*<0.05) (Figure 2E,F).

The article "The potency of lncRNA MALAT1/miR-155/CTLA4 axis in altering Th1/Th2 balance of asthma" was retracted in 2023. Reasons: duplicated images; concerns about the images.

**Figure 2:** The *in-vitro* impacts of MALAT1 and miR-155 on Th1/Th2 and T-bet/GATA3 ratios (**A**) The expression of MALAT1 was evaluated after respective transfection of pcDNA3.1-MALAT1, si-MALAT1-1, si-MALAT1-2, si-MALAT1-3 and si-MALAT1-1 into CD^4+^ T cells. *: *P*<0.05 when compared with NC. (**B**) The expression of miR-155 within CD^4+^ T cells was determined when miR-155 mimic and miR-155 inhibitor were transfected. *: *P*<0.05 when compared with miR-NC. (**C**) The mRNA levels of IFN-γ, IL-2 and T-bet were determined within CD^4+^ T cells of pcDNA3.1-MALAT1, si-MALAT1-3, miR-155 mimic and miR-155 inhibitor groups. *: *P*<0.05 when compared with NC. (**D**) The protein levels of IFN-γ, IL-2 and T-bet were appraised within CD^4+^ T cells transfected by pcDNA3.1-MALAT1, si-MALAT1-3, miR-155 mimic and miR-155 inhibitor. *: *P*<0.05 when compared with NC. (**E**) The mRNA levels of IL-4, IL-10 and GATA3 were contrasted among cells transfected with pcDNA3.1-MALAT1, si-MALAT1-3, miR-155 mimic and miR-155 inhibitor. *: *P*<0.05 when compared with NC. (**F**) The protein levels of IL-4, IL-10 and GATA3 within CD^4+^ T cells were detected among pcDNA3.1-MALAT1, si-MALAT1-3, miR-155 mimic and miR-155 inhibitor groups. *: *P*<0.05 when compared with NC.

### MALAT1 modulated expression of miR-155 by sponging it

The binding sites of MALAT1 and miR-155 were predicted through usage of starBase software (http://starbase.sysu.edu.cn/), and pRL-TK/Rluc-MALAT1 Wt co-transfected with miR-155 mimic profoundly attenuated the luciferase activity of CD^4+^ T cells in comparison with RL-TK/Rluc-MALAT1 Mut+miR-155 mimic group and RL-TK/Rluc-MALAT1 Wt+miR-NC group (*P*<0.05) (Figure 3A). Moreover, silencing of MALAT1 could strongly up-regulate the expression of miR-155 (*P*<0.05), whereas over-expressed MALAT1 reduced miR-155 expression (*P*<0.05) (Figure 3B). Nonetheless, the expression of MALAT1 stayed stable within CD^4+^ T cells no matter whether miR-155 was over-expressed or under-expressed (*P*<0.05) (Figure 3B).

**Figure 3:** The regulatory relationships among MALAT1, miR-155 and CTLA-4 within CD^4+^ T cells (**A**) The luciferase activity of CD^4+^ T cells was monitored among pRL-TK/Rluc-MALAT1 Wt+miR-155 mimic, pRL-TK/Rluc-MALAT1 Mut+miR-NC and pRL-TK/Rluc-MALAT1 Mut+miR-155 mimic groups. *: *P*<0.05 when compared with pRL-TK/Rluc-MALAT1+miR-NC. (**B**) The miR-155 expression was detected after transfection of pcDNA3.1-MALAT1 or si-MALAT1-3, and the expression of MALAT1 was measured under treatment of miR-155 mimic or miR-155 inhibitor. *: *P*<0.05 when compared with NC/miR-NC group. (**C**) The luciferase activities of CD^4+^ T cells in the pRL-TK/Rluc-CTLA-4 Wt+miR-155 mimic, pRL-TK/Rluc-CTLA-4 Mut+miR-NC and pRL-TK/Rluc-CTLA-4 Mut+miR-155 mimic groups were compared. *: *P*<0.05 when compared with pRL-TK/Rluc-CTLA-4+miR-NC. (**D**) The expression of CTLA-4 was measured after transfection of miR-155 mimic and miR-155 inhibitor into CD^4+^ T cells. *: *P*<0.05 when compared with NC. (**E**) The CTLA-4 expression was assessed within CD^4+^ T cells transfected by pcDNA3.1-CTLA-4, si-CTLA-4-1, si-CTLA-4-2 and si-CTLA-4-3. *: *P*<0.05 when compared with NC. (**F**) The expression of miR-155 was modified when pcDNA3.1-CTLA-4 and si-CTLA-4-1 were transfected, respectively. *: *P*<0.05 when compared with NC.

The article "The potency of lncRNA MALAT1/miR-155/CTLA4 axis in altering Th1/Th2 balance of asthma" was retracted in 2023. Reasons: duplicated images; concerns about the images.

### CTLA-4 interfered with the impacts of miR-155 and MALAT1 on Th1/Th2 balance and T-bet/Gata3 ratio within CD^4+^ T cells

The binding sites between miR-155 and CTLA-4 were speculated based on miRBase software (http://www.mirbase.org/) (Figure 3C). And cells treated by pRL-TK/Rluc-CTLA-4 Wt+miR-155 mimic exhibited a lower luciferase activity than those treated with pRL-TK/Rluc-CTLA-4 Wt+miR-NC or by pRL-TK/Rluc-CTLA-4 Mut+miR-155 mimic (both *P*<0.05). Additionally, expression of CTLA-4 was cut down markedly under the influence of miR-155 mimic (*P*<0.05), yet miR-155 inhibitor increased CTLA-4 expression in the CD^4+^ T cells (*P*<0.05) (Figure 3D).

Moreover, though pcDNA3.1-CTLA-4 triggered a rise of CTLA-4 expression within CD^4+^ T cells, si-CTLA-4 (i.e. si-CTLA-4-1, si-CTLA-4-2 and si-CTLA-4-3) tended to decrease the expression of CTLA-4 (*P*<0.05) (Figure 3E). Given an optimum efficacy of si-CTLA-4-1 in down-regulating CTLA-4 expression, it was thus recommended as an inhibitor of CTLA-4 expression in the following cellular experiments. However, the expression of miR-155 was not altered, when pcDNA3.1-CTLA-4 and si-CTLA-4-1 was transfected (*P*>0.05) (Figure 3F).

Furthermore, miR-155 mimic could substantially elevate the protein/mRNA levels of Th1-type cytokines (i.e. IFN-γ and IL-2) and T-bet in comparison with the pcDNA3.1-CTLA-4+miR-155 mimic group (*P*<0.05) (Figure 4A,C). Conversely, the protein/mRNA levels of Th2-type cytokines (i.e. IL-4 and IL-10) and GATA3 descended in the miR-155 mimic group (*P*<0.05) (Figure 4B,D). With respect to MALAT1, its expressional change could alter CTLA-4 expression observably (*P*<0.05) (Figure 5A), but CTLA-4 expression failed to modify the expression of MALAT1 (*P*>0.05) (Figure 5B). Furthermore, when compared with si-MALAT1-3 group, pcDNA3.1-CTLA-4 combined with si-MALAT1-3 led to an expressional reduction of Th1-type cytokines (i.e. IFN-γ and IL-2) and T-bet, while mRNA and protein levels of Th2-type cytokines (i.e. IL-4 and IL-10) and GATA3 were enhanced under the treatments (*P*<0.05) (Figure 5C–F).

The article "The potency of lncRNA MALAT1/miR-155/CTLA4 axis in altering Th1/Th2 balance of asthma" was retracted in 2023. Reasons: duplicated images; concerns about the images.

**Figure 4:** The interference effect of CTLA-4 on the contribution of miR-155 to Th1/Th2 and T-bet/GATA3 ratios within CD^4+^ T cells (**A**) The mRNA levels of IFN-γ, IL-2 and T-bet within CD^4+^ T cells were monitored among pcDNA3.1-CTLA-4+miR-155 mimic, miR-155 mimic and NC groups. *: *P*<0.05 when compared with NC group. (**B**) The mRNA levels of IL-4, IL-10 and GATA3 were examined within CD^4+^ T cells of pcDNA3.1-CTLA-4+miR-155 mimic, miR-155 mimic and NC groups. *: *P*<0.05 when compared with NC. (**C**) The protein levels of IFN-γ, IL-2 and T-bet were detected among CD^4+^ T cells of pcDNA3.1-CTLA-4+miR-155 mimic, miR-155 mimic and NC groups. *: *P*<0.05 when compared with NC. (**D**) The protein levels of IL-4, IL-10 and GATA3 were determined within CD^4+^ T cells of pcDNA3.1-CTLA-4+miR-155 mimic, miR-155 mimic and NC groups. *: *P*<0.05 when compared with NC.

**Figure 5:** The contribution of CTLA-4 to hindering the impacts exerted by si-MALAT1-3 on Th1/Th2 and T-bet/GATA3 balances within CD^4+^ T cells (**A**) Expression of CTLA-4 was subjected to regulation of pcDNA3.1-MALAT1 and si-MALAT1-3. *: *P*<0.05 when compared with NC. (**B**) The expression of MALAT1 remained stable under the transfection of pcDNA3.1-CTLA-4 or si-CTLA-4-1. *: *P*<0.05 when compared with NC. (**C**) The mRNA levels of IFN-γ, IL-2 and T-bet within CD^4+^ T cells were compared among pcDNA3.1-CTLA-4+si-MALAT1-3, si-MALAT1-3 and NC groups. *: *P*<0.05 when compared with NC group. (**D**) The mRNA levels of IL-4, IL-10 and GATA3 were drawn from CD^4+^ T cells transfected by pcDNA3.1-CTLA-4+si-MALAT1-3, si-MALAT1-3 and NC. *: *P*<0.05 when compared with NC. (**E**) The protein levels of IFN-γ, IL-2 and T-bet were obtained from CD^4+^ T cells transfected by pcDNA3.1-CTLA-4+si-MALAT1-3, si-MALAT1-3 and NC. *: *P*<0.05 when compared with NC. (**F**) The protein levels of IL-4, IL-10 and GATA3 were determined among pcDNA3.1-CTLA-4+si-MALAT1-3, si-MALAT1-3 and NC groups. *: *P*<0.05 when compared with NC.

## Discussion

Airway inflammation induces reversible airway obstruction and airway hyper-responsiveness, which are key asthma features. The CD^4+^ T cells are major participators in asthma-relevant inflammation [39], and the skewing of T cells into Th2 cells causes an imbalance of Th1-type and Th2-type cytokines, which promotes the onset and progression of asthma [40,41]. Since the transcription factors, such as T-bet and GATA-3, enhance the production of Th1-type cytokines (e.g. IFN-γ) [42] and Th2-type cytokines (e.g. IL-4 and IL-5), respectively [43], the T-bet/GATA3 ratio investigated here (Figure 1E) are viewed as a reflection of Th1/Th2 balance [44]. Based on the findings, the Th1/Th2 balance and T-bet/GATA3 ratio that varied within CD^4+^ T cells appeared as reliable indicators of asthma progression, and in this investigation we focused on them as markers of dysregulated inflammation underlying asthma etiology.

The article "The potency of lncRNA MALAT1/miR-155/CTLA4 axis in altering Th1/Th2 balance of asthma" was retracted in 2023. Reasons: duplicated images; concerns about the images.

Our results showed that both the Th1/Th2 ratio and the T-bet/GATA3 ratio were markedly reduced within asthma patients when compared with healthy controls (Figure 1B and Table 2), and there were negative correlations between MALAT1 expression and these ratios (Figure 1C). We partly ascribed this association to the fact that up-regulated MALAT1 expression could enable production of Th2-type cytokines and simultaneously curb release of Th1-type cytokines by CD^4+^ T cells (Figure 2). Actually, the role of MALAT1 in modulating inflammation, though hidden, has been implicated before. For instance, over-expressed MALAT1 was found to increase expression of p38 MAPK and NF-κB [19], whose activities were intensified in mice models of asthma [45,46]. Beyond that, p38 MAPK and NF-κB both could boost production of asthma-related cytokines, including IL-1β, IL-4, IL-5, IL-6 and IL-13 [47–49]. Besides, macrophages tended to display M2-like traits under the guidance of MALAT1, which was manifested by over-expressed IL-12 and under-expressed TNF-α, IL-6 and IL-10 [22,50]. Drawing on these findings, the current study established a link between MALAT1 and Th1/Th2 imbalance-triggered inflammation, which was also validated in asthma cell models here (Figure 2).

Our findings also showed that MALAT1 was capable of negatively modulating miR-155 expression in CD^4+^ T cells by sponging it (Figure 3A,B), just as in glioma [26]. These findings demonstrated that MALAT1 regulated asthmatic inflammation by targeting miR-155. In fact, miR-155 modified inflammation-related pathways (e.g. MAPK signaling [51] and JAK-STAT signaling [52]), and transcriptional activation of bic, from which the transcription product of miR-155 derived, was capable of activating T cells [53]. Despite consensus on the tight linkage of miR-155 with T cell-induced inflammation, Malmall et al. held that knockout of miR-155 tended to ease asthma development in mice models [28], which conflicted with the results of this study (Figure 1D). We strived to explain this divergence from following two aspects. In the first place, the asthma mice models adopted by Malmall et al. were established based on induction of OVA, yet the asthma patients we recruited were affected by non-uniform allergens [28]. The diversified pathogens could bring about inconsistent biological actions inside’. different types of organisms, along with discrepant expressional profiles of miRNAs. Second, the incorporated asthma patients, albeit in a relatively large scale, were not subdivided according to living habits here, which might overlook the impact of environmental parameters on miR-155 expression. Another noteworthy point of the present study lied in that MALAT1 affected expression of Th1-type and Th2-type cytokines more strongly than miR-155 (Figure 2), which could be ascribed to that MALAT1 might sponge and modify other asthma inflammation-relevant miRNAs. For instance, miR-206, miR-299-5p and miR-126, which were potentially sponged by MALAT1 (http://starbase.sysu.edu.cn/agoClipRNA.php?source=lncRNA), were sensitive biomarkers for asthma of various severities [20]. Nonetheless, intensive exploration should be carried out to validate the contribution of MALAT1 and the abovementioned miRNAs to asthmatic inflammation.

The article "The potency of lncRNA MALAT1/miR-155/CTLA4 axis in altering Th1/Th2 balance of asthma" was retracted in 2023. Reasons: duplicated images; concerns about the images.

Of note, CTLA-4 altered the modulatory effects of MALAT1 and miR-155 on Th1/Th2 balance and T-bet/GATA3 ratio in CD^4+^ T cells (Figures 4 and 5). In practice, the relationship of CTLA-4 and T-cell activity were intertwined. For example, CTLA-4 could stagnate the cell cycle of activated T cells by blocking CD28-inducing reactions and reducing IL-2 expression [54]. Moreover, CTLA-4 combined with B7-1 and B7-2 might aid to maintain peripheral tolerance of T cells [55,56], and elevating CTLA-4 expression could facilitate differentiation of Th0 cells into early-stage Th2 cells [57]. Apart from that, the CTLA-4 also presented a negative feedback effect against aggravated inflammation [58,59], which suggested that the failure to sustain high CTLA-4 expression might make asthmatics unable to suppress Th2-cell differentiation. Adding to these prior observations, our study shows for the first time that CTLA-4 regulates asthma inflammation by modifying the effects of MALAT1 and miR-155 (Figures 3D and 5A).

In conclusion, our study indicates that MALAT1 sponging miR-155 could alter the Th1/Th2 balance within CD^4+^ T cells through a CTLA-4-dependent mechanism. Further studies are needed to determine whether targeting the MALAT1/miR-155/CTLA-4 axis could alter the Th2 responses that promote airway inflammation in asthma.

## Abbreviations

ASM: airway smooth muscle
CTLA4: CTL-associated antigen 4
EDTA: ethylene diamine tetraacetic acid
FeNO: fractional exhaled nitric oxide
FEV1: forced expiratory failure volume in 1 s
FVC: forced vital capacity
GAPDH: glyceraldehyde-3-phosphate dehydrogenase
GATA3: GATA-binding protein 3
IFN: Interferon
MACS: magnetic activated cell sorting
MALAT1: metastasis-associated lung adenocarcinoma transcript 1
OVA: ovalbumin
PBMC: peripheral blood mononuclear cell
PBS: phosphate buffer solution
RT-PCR: reverse transcription-polymerase chain reaction
Th: T helper
Treg: regulatory T cell
Wt: wild-type
